The article "Lung Diseases Detection Using Various Deep Learning Algorithms" was published in 2023. Journal: J Healthc Eng.

# Lung Diseases Detection Using Various Deep Learning Algorithms

**DOI:** 10.1155/2023/3563696

**Published:** 2023-02-03

**Authors:** M. Jasmine Pemeena Priyadarsini, Ketan kotecha, G. K. Rajini, K. Hariharan, K. Utkarsh Raj, K. Bhargav Ram, V. Indragandhi, V. Subramaniyaswamy, Sharnil Pandya

**Affiliations:** ^1^School of Electronics Engineering, Vellore Institute of Technology, Vellore 632014, India; ^2^Symbiosis Centre for Applied Artificial Intelligence, Symbiosis International (Deemed University), Pune, India; ^3^School of Mathematical Sciences, Sunway University, Subang Jaya, Malaysia; ^4^School of Electrical Engineering, Vellore Institute of Technology, Vellore 632014, India; ^5^School of Computing, SASTRA Deemed University, Thanjavur, India; ^6^Computer Science and Media Technology Department, Faculty of Technology, Linnaeus University, P G Vejdes väg 351 95, Växjö, Sweden

## Abstract

The primary objective of this proposed framework work is to detect and classify various lung diseases such as pneumonia, tuberculosis, and lung cancer from standard X-ray images and Computerized Tomography (CT) scan images with the help of volume datasets. We implemented three deep learning models namely Sequential, Functional & Transfer models and trained them on open-source training datasets. To augment the patient's treatment, deep learning techniques are promising and successful domains that extend the machine learning domain where CNNs are trained to extract features and offers great potential from datasets of images in biomedical application. Our primary aim is to validate our models as a new direction to address the problem on the datasets and then to compare their performance with other existing models. Our models were able to reach higher levels of accuracy for possible solutions and provide effectiveness to humankind for faster detection of diseases and serve as best performing models. The conventional networks have poor performance for tilted, rotated, and other abnormal orientation and have poor learning framework. The results demonstrated that the proposed framework with a sequential model outperforms other existing methods in terms of an F1 score of 98.55%, accuracy of 98.43%, recall of 96.33% for pneumonia and for tuberculosis F1 score of 97.99%, accuracy of 99.4%, and recall of 98.88%. In addition, the functional model for cancer outperformed with an accuracy of 99.9% and specificity of 99.89% and paves way to less number of trained parameters, leading to less computational overhead and less expensive than existing pretrained models. In our work, we implemented a state-of-the art CNN with various models to classify lung diseases accurately.

The article "Lung Diseases Detection Using Various Deep Learning Algorithms" was published in 2023. Journal: J Healthc Eng.

## 1. Introduction

Lungs play a vital role in the human system, which performs expansion and relaxation to bring in oxygen and take out carbon dioxide. Lung diseases are respiratory diseases that affect the various organs and tissues associated with breathing, leading to airway diseases, lung tissue diseases, and lung circulation diseases. Some of the respiratory diseases like common cold and influenza cause mild discomfort and hindrance while others like pneumonia, tuberculosis and lung cancer are life-threatening and cause severe acute respiratory problems [1].

According to a research study done by the Forum of International Respiratory Societies called “The Global Impact of Respiratory Disease,” 10.4 million people suffered mild or severe symptoms of tuberculosis, and 1.4 million of those affected died as per the survey reported [2]. Lung cancer kills an astounding number of people every year. More than 1.6 million people were reported to have died in the year the survey was carried out. Pneumonia is one of the top respiratory diseases and 1.23 million children under the age of 5 died due to pneumonia according to the Johns Hopkins Bloomberg School of Public Health report titled “Pneumonia and Diarrhea Progress Report 2020” [3]. Detection of the abovementioned diseases at the early stages of infection can drastically increase the chances of survival and can prevent human casualities. Chest X-ray images and CT scans are common examinations that determine the presence of these diseases [4]. The presence of trained professionals is required to examine the scanned images and determine the infections. According to the Union Health Ministry data statistics there exists a shortfall of 76.1 percent of physicians at the Community Health Centres (CHCs) in rural areas. To overcome this, deep learning techniques are implemented, which pave the way for a new strategy.

Deep learning is a branch of machine learning that provides state-of-the-art accuracy and is a subset of the artificial intelligence with representation learning. This tool has drawn attention in recent times due to their ability to read image data, process them, and provide results based on the previously trained data [5]. Deep learning models can learn features and patterns from dataset images and use the learned features to classify new test images that have not been previously visualized by the model.

Numerous works have already been conducted by researchers around the world and have led to promising results. These works can help support existing methods or open pathways to new ones that could not have been possible. These advancements can help in quick and accurate detection as well as classification of diseases and provide quick support to obtain impressive results to eliminate deadly infectious diseases.

The article "Lung Diseases Detection Using Various Deep Learning Algorithms" was published in 2023. Journal: J Healthc Eng.

The rest of the manuscript is structured as follows: In Section 2, we introduce the basic foundation of the convolution neural networks.  Section 3 describes the architecture of the proposed model.  Section 4 discusses the implementation of the proposed CNN technique and the experimental results. Finally, we conclude our work with a summary and future directions in Section 5.

## 2. Related Work

One of the best techniques currently used in medical image analysis are CNNs, which have a remarkable efficiency in classifying the images. Some of the contemporary CNN models are Pre-Trained, Functional, and Sequential, which are reviewed in the forthcoming sections.

Liu et al. proposed three different types for the applications of CNN-trained models in tuberculosis detection. In all these three methods, features are extracted by the CNN architectures and are trained by the support vector machine (SVM), and in the second proposal, features are extracted from coreference resolution (CR) and are trained in the SVM classifier. In the third proposal, these two proposals are combined together to create an ensemble of the classifiers. The Montgomery dataset has a total of 138 X-ray images and the Shenzhen dataset has a total of 662 X-ray images. These trained models help reduce the processing time but provide low accuracy, which is not conducive and cannot be implemented in medical diagnosis.

Amit Kumar Jaiswal, Prayag Tiwari, Sachin Kumar, and Deepak Gupta proposed a method called mask RCNN. It is a deep neural network model that can extract two types of features: global and local. Pixel-wise division is carried out and this method is expected to have a better performance evaluated on the radiograph dataset. This technique highlights the infected regions and provides a heat map for better understanding for people looking at the results. But they have ensembled ResNet50 and ResNet101 (Mask RCNN models) but achieved less biased results than expected and require more GPU processing power to train.

Elshennawy and Ibrahim, presented on four different models. Among these four models, CNN and LSTM-CNN started from the beginning and the other two are pretrained models and the specific models used are ResNet152v2 and MobileNetV2. They formulated to create from the ground, a deep learning neural network model, which could diagnose pneumonia symptoms using chest X-ray images, which has pneumonia [6]. Some of the disadvantages are that it has a humongous architecture with hundreds of millions of trainable parameter weights [7, 8]. This type of model requires high computing and processing power.

The article "Lung Diseases Detection Using Various Deep Learning Algorithms" was published in 2023. Journal: J Healthc Eng.

Various deep learning techniques, Naik and Edla [9] developed a lung nodule classification and identification model for computed tomography (CT) images. The CT scans required a computer-aided detection system for categorizing the lung nodule into benign and malignant types, along with the highest level of accuracy to protect from a delay in diagnosis. The deep learning approaches used to categorize the lung nodule have positive outcomes compared to other methods. When the mutations were implemented in the deep learning architecture, the accuracy of the classification system increased rapidly. The deep learning method was used to specify the new impacts in nodule classification and also recognized the preliminary stage of a malignant lesion [10].

## 3. Proposed Methodology

This section discusses the datasets used, the preprocessing, the data augmentation methods, and the various algorithms used. The workflow of the proposed technique is presented in a flowchart form in Figure 1.

### 3.1. Datasets

All the datasets used in this work are from opensource datasets published on the website “Kaggle.”

The pneumonia dataset published by Paul Mooney contains 5,856 frontal chest X-ray images, 1,583 images of the dataset are of people with no abnormalities in their lungs, and 4,273 images predict some abnormalities and symptoms of pneumonia.

The tuberculosis dataset published by Scott Mader has 662 frontal X-rays. These images were collected by physicians in the Guangdong Hospital, Shenzhen, China. Hence, this dataset is commonly known as the Shenzhen dataset. It contains 326 images, which contains lung images of healthy persons and in turn contains 336 images that are infected by tuberculosis.

The cancer dataset published by Mohamed Hany has 907 lung CT-scan images, 215 images of the dataset are of people with no signs of cancer, and 692 images of the dataset are of people with cancer. The dataset contains 3 types of cancer images: adenocarcinoma, large cell carcinoma, and squamous cell carcinoma.  Figure 2 shows few sample images from the CT-scan dataset.

#### 3.1.1. Preprocessing and Data Augmentation

The images present in the datasets are of different resolutions. However, the CNN models require images to be of one specified size. Hence, all the images in the dataset were resized to 224 × 224. Lowering the input image size helps process a faster execution of images and thus, makes the model faster for the specific associated task.

Data augmentation is a common support method used to significantly increase the training data volume by introducing slight variations of an image in each training epoch. The variations used in this work are horizontal flip, zoom, shear, rotation, and rescale. This technique is essential to get high levels of accuracy as the CNN model is able to train on more data than originally present in the dataset.  Figure 3 shows the variations that can be created from one sample image.

The article "Lung Diseases Detection Using Various Deep Learning Algorithms" was published in 2023. Journal: J Healthc Eng.

### 3.2. Deep Learning Algorithms

In recent times, a dataset of medical images has been available in the Kaggle repository. In this paper, this dataset has been implemented using the novel models of CNN, namely, sequential and functional models, combining CNN and data augmentation. Three different model algorithms were deployed in this proposed work. These are explained in detail in the following subsections.

#### 3.2.1. Sequential Model

The sequential model is a model in which layers are stacked to form a sequential order. The input is passed through all the layers in the order in which the layers are stacked. Features are learnt at each and every layer and more deeper into the layer, the model is capable of distinguishing the infected areas and noninfected areas from the chest X-rays [11].

The proposed sequential model has five convolutional layers with the number of filters increasing as it proceeds deeper into the network [12]. The alpha parameter was set to 0.66. Leaky ReLU allows a small gradient to pass through, while ReLU completely removes any gradient when the unit is not active. In addition, max pooling was carried out after each activation. Adam optimizer and learning rate of 0.0001 was employed. The block diagram of the sequential model is presented in Figure 4.

#### 3.2.2. Functional Model

The functional model has more flexibility than the other algorithms. It can form connections between any two layers contrary to the others and progress in a linear fashion. This allows us to create more complicated and sophisticated networks [13]. The input goes through the first layer and then proceeds along the designed architecture. This method also trains from the beginning, contrary to the pretrained model.

The proposed functional model has two convolution layers of 7 × 7 window and another with 1 × 1 on top of 3 × 3 window as presented in Figure 5. The input is passed through both convolution layers separately and then the output from both layers is appended and then passed to five 3 × 3 convolution layers. The Adam optimizer with learning rate = 0.0001 was employed.

#### 3.2.3. Pretrained Model

This is the easiest and most commonly used model for image classification. Instead of training a model from the beginning, this technique uses already trained weights on a large dataset of images to classify the required images [14, 15]. This technique is also called transfer learning as previously learned weights are transferred and used for classification. Generally, this model takes less time to train and produces better results and accuracy.

The article "Lung Diseases Detection Using Various Deep Learning Algorithms" was published in 2023. Journal: J Healthc Eng.

The pretrained model used here is VGG-16, a convolutional neural network (CNN), famous for high accuracy and achieved the top 5 accuracies in the ImageNet competition with an accuracy of 97.7%.

## 4. Results and Discussion

The various models were trained, their accuracies and losses were plotted, and the test accuracy was obtained and compared with other research works for lung disease detection with CNN [16, 17]. The performance metrics involved in this proposed work are accuracy, precision, recall, and F1 score.

(i) Accuracy represents the number of correctly classified data instances over the total number of data instances.
  (1) $$\begin{array}{c} Accuracy=\frac{TP+TN}{TP+TN+FP+FN}\text{,} \end{array}$$
  where, true positive is abbreviated as TP, true negative as TN, false positive as FP, and false negative as FN.
(ii) Precision should ideally be 1 (high) for a good classifier. Precision becomes 1 only when the numerator and denominator are equal, i.e, TP = TP + FP, this also means FP is zero. As FP increases, the value of the denominator becomes greater than the numerator and the precision value decreases.
  (2) $$\begin{array}{c} precision=\frac{TP}{TP+FP}\text{.} \end{array}$$
(iii) Recall is also known as sensitivity or true positive rate and is defined as follows:
  (3) $$\begin{array}{c} Recall=\frac{TP}{TP+FN}\text{.} \end{array}$$
(iv) F1-score is a metric that takes into account both precision and recall and is defined as follows:
  (4) $$\begin{array}{c} F1\;score=2*\frac{precision*Recall}{precision+Recall}\text{.} \end{array}$$

### 4.1. Sequential Model for Pneumonia

In medical diagnostics, it is common to analyze the classifier performance using sensitivity (true positive rate) and specificity (true negative rate) instead of accuracy [6]. To assess the overall classification F1 score is computed [7, 18]. From the dataset of 5,856 chest X-ray images, 2,000 images were used for training of which 1,000 images were of normal chest X-rays and the other 1,000 images were of pneumonia-infected chest X-rays.

The model was trained for 50 epochs.  Figure 6 shows the increase in accuracy as the model trains with trained set images and Figure 7 shows that the loss encountered with this model is less. The accuracy starts from 75% and gradually increases to 90% with 10 epochs.

After training, the model was used to predict the labels of test images that were not known by the model during training. The test image set had 583 images of normal chest X-rays and 3,273 images of pneumonia-infected chest X-rays.  Table 1 provides accuracy of our model with the existing works related to pneumonia and found that our model outperforms other existing works. The model predicted the labels accurately for 533 images from 583 normal CXR images and 3,070 images from 3,273 pneumonia-infected CXR images.

The article "Lung Diseases Detection Using Various Deep Learning Algorithms" was published in 2023. Journal: J Healthc Eng.

### 4.2. Sequential Model for Tuberculosis

The tuberculosis dataset has a grand total of 662 chest X-ray images. Among 662 images, 285 images of normal chest X-rays and 292 images of tuberculosis-infected chest X-rays were used for training. As depicted in Figure 8, the tuberculosis model started with a very low accuracy of 50%. After training for around 100 epochs, the model accuracy value of 97% was obtained.

Numerous works have already been carried out by researchers around the world and have led to promising results. These works can help support the existing methods or open pathways to new methods, which could not have been possible before [8, 24]. These advancements can help in faster and accurate detection, as well as classification of diseases and provide support to obtain impressive results to eliminate deadly infectious diseases.

The model was used to predict the labels for test images. The test image set had a total of 85 images of which 41 were of normal and 44 were of tuberculosis-infected. The model predicted 37 images of normal and 39 images of tuberculosis-infected accurately as presented in Figure 9.  Table 2 provides an accuracy of our model with existing works related to tuberculosis and finds to be superior when compared to other existing works.

### 4.3. Functional Model for Cancer

The dataset has a total of 907 lung CT-scan images, 215 images of people with no signs of cancer, and 692 images of people infected with cancer were used for training the model [30, 31]. The model was trained for 100 epochs. As seen in Figure 10, the model started with an accuracy of 70% and increased to 90% in about 10 epochs.

The model was presented to predict for the test images. The test dataset had a total of 278 images, of which 224 were cancer infected and 54 were normal. The model accurately predicted 54 images of normal and 204 images of cancer infected, and the loss is shown in Figure 11.

Table 3 depicts the accuracy of our model with existing works related to cancer and finds to be extraordinary when compared to other existing works.

### 4.4. Functional Model for Pneumonia

The dataset used for the functional model is the one that was utilized in sequential model. The model accuracy starts from around 81% and rapidly increases to 90% in less than 5 epochs.

### 4.5. Pretrained Model for Pneumonia

Figure 12 shows the model accuracy gradual improvement for the pneumonia disease with the functional model. The same dataset was used for this model, i.e., from Paul Mooney with 5,856 images of which 1,000 are normal X-rays and other 1,000 are infected chest X-rays. As the model has already been trained before, the starting accuracy is very good. There is a minor improvement after training for 15 epochs as is evident in Figure 13.

The article "Lung Diseases Detection Using Various Deep Learning Algorithms" was published in 2023. Journal: J Healthc Eng.

Figure 14 shows that the initial model loss is low as compared to the other models, hence, there is no continuous progress like that in the sequential and functional models.

Figure 15 shows that the pretrained models are easy to train and that the loss gradually decreases as they have previously been trained on various datasets.

## 5. Conclusion and Future Work

We have proposed three different architecture models of CNNs, which were used to train on various lung diseases that are available in the open-source dataset. The trained models were used to predict the labels of some test images that were not visualized by the models. The results of the proposed models performed better than other related works. The results obtained through this framework with a sequential model outperform other existing methods in terms of F1 score, accuracy and recall for pneumonia and for tuberculosis. In addition, the functional model for cancer outperformed with accuracy and specificity, and it requires less computation cost and time. In future, varying the optimizers, learning rate, and introduction of more data augmentation could potentially lead to further improvements in the classification accuracy of the proposed CNN models. Early stopping techniques will likely provide further insights into diagnosing lung diseases that can be passed down to avoid overfitting.

## Figures and Tables

**Figure 1:** Workflow of the classification model.

**Figure 2:** Chest-CT scan images (source: kaggle).

**Figure 3:** Variations of a chest X-ray image.

**Figure 4:** Block diagram of sequential model.

**Figure 5:** Block diagram of functional model.

**Figure 6:** Model accuracy vs. epochs for pneumonia (sequential).

**Figure 7:** Model loss vs. epochs for pneumonia (sequential).

**Figure 8:** Model accuracy vs. epochs for tuberculosis.

**Figure 9:** Model loss vs. epochs for tuberculosis.

**Figure 10:** Model accuracy vs. epochs for cancer.

**Figure 11:** Model loss vs. epochs for cancer.

**Figure 12:** Model accuracy vs. epochs for pneumonia (functional).

**Figure 13:** Model loss vs. epochs for pneumonia (functional).

**Figure 14:** Model accuracy vs. epochs for pneumonia (pretrained).

**Figure 15:** Model loss vs. epochs for pneumonia (pretrained).

The article "Lung Diseases Detection Using Various Deep Learning Algorithms" was published in 2023. Journal: J Healthc Eng.

**Table 1:** Comparison of our model with existing works related to pneumonia.

Related work	Dataset	Techniques	F1score	Accuracy	Recall	Precision	Specificity
Sourab and Kabir [19]	Mendeley datav2 (5856 images)	CNN	96	94.55	94	99	85
Gayathri [20]	GitHub (783 images)	CNN	95.63	95.78	—	95.63	95
Vrbančič and Podgorelec [21]	ImageNet	Ensemble	95.01	91.98	93.8	96.38	90
Fernandes et al. [22]	CXR dataset (3883 images)	CNN	93.2	95.7	91.2	95.1	97.5
Hasija et al. [23]	—	CNN	98.52	98.38	—	—	99.81
Our proposed model	Chest X-ray (1000 images)	CNN-sequential model	98.55	98.4375%	96.33%	99%	99.89%

**Table 2:** Accuracy of our model with existing works related to tuberculosis.

Authors	Dataset	Techniques	F1-score	Accuracy	Recall	Precision
Momeny et al. [25]	Annotated (1078 images)	CNN	89	93	85	92
Lopes and Valiati [26]	ImageNet (10000 images)	CNN	—	76	—	—
Sineglazov et al. [27]	National institute of phthisiology and pulmonology (9311 slices)	CNN	99.04	99	97.6	98.34
Mamalakis et al. [28]	CXR dataset (3883 images)	ResNet CNN	81.64	71	91	78.6
Duong et al. [29]	(i) Montgomery county & CXR dataset (138 images) (ii) Shenzhen dataset (662 images)	CNN	97.9	99	—	—
Our proposed model	Chest X-ray (662 images)	CNN	97.99	99.4%	98.8	98.55

**Table 3:** Accuracy of our model with existing works related to cancer.

Authors	Dataset	Techniques	Accuracy	Specificity	Sensitivity
Lee et al. [32]	Annotated dataset-87	CNN	92.5	—	—
Tomassini et al. [33]	Planar data	CNN	74	—	81%
Wei et al. [34]	Annotated dataset-500 images	CNN	99.3	98.31	100
Desai and Shah [35]	Annotated dataset-1000 images	MLP	91.92	92.3	91
Hassantabar et al. [36]	Annotated dataset-682 images	CNN	93.20	99.71	96.09
Our proposed model	278 images	CNN	99.9	99.89	100

## Data Availability

The data used to support the findings of this study are available from the corresponding author upon request.
